# Prediction Effect of Amplitude-Integrated EEG on the Brain Damage and Long-Term Nervous System Development of Late Preterm Infants

**DOI:** 10.1155/2021/4041082

**Published:** 2021-09-23

**Authors:** Sehua Qu, Lianqiang Shan, Zhen Zhang, Wansheng Peng, Yun Chen, Hui Zhang, Huaifu Dong, Xin Chen

**Affiliations:** ^1^Department of Pediatrics, The First Affiliated Hospital of Bengbu Medical College, Bengbu, Anhui 233000, China; ^2^Department of Pediatrics, The Second Affiliated Hospital of Bengbu Medical College, Bengbu, Anhui 233000, China

## Abstract

In order to explore the prediction effect of amplitude-integrated EEG on the brain damage and long-term nervous system development of late preterm infants, this paper uses the hospital's late preterm infants as the research object and analyzes the prediction effect of amplitude-integrated EEG on the brain damage and long-term nervous system development of late preterm infants through controlled trials. Among them, the test group used amplitude-integrated EEG for prediction analysis, and the control group used traditional clinical prediction methods. Furthermore, the real-time monitoring and short-term prediction effects of amplitude-integrated EEG on brain damage in late preterm babies and the prediction impact on long-term nervous system development are evaluated in this study. It incorporates statistical techniques to evaluate the findings statistically. In addition, a nonparametric rank-sum test is used in this work, and a chi-square test is used to compare enumeration data across groups. Through experimental research, it can be seen that the amplitude-integrated EEG has a pronounced prediction effect on the brain damage and long-term nervous system development of late preterm infants, and the effect is higher than that of the traditional clinical prediction methods.

## 1. Introduction

Amplitude-integrated EEG is a new type of EEG monitoring technology, which aims to analyze EEG through the amplitude waves of EEG signals. Amplitude-integrated EEG can monitor the neurophysiological activities of children within 6 hours of birth and intuitively reflect the changes of EEG background activities and epileptiform activities. Moreover, it can realize bedside monitoring and has many advantages such as convenient operation, noninvasive, intuitive graphics, and easy analysis. However, because preterm infants are more sensitive to infection, hypoxia, ischemia, and inflammation, the risk of brain damage is also higher. In severe cases, it may even threaten the life of preterm infants [1]. To successfully reduce preterm baby mortality and enhance their quality of life, it is essential to establish EEG monitoring in time for preterm babies, identify their brain damage symptoms as soon as feasible, implement treatments as soon as possible, and conduct prognosis evaluations [2].

aEEG is a simplified method of monitoring the electrical activity of the cerebral cortex. It can monitor the neuroelectrophysiological activity in children's early postnatal period, reflect the changes in the background activity of the brain electrical activity and epileptiform activities, and improve the early diagnosis and prognostic evaluation of brain injury. In the current clinical experimental studies, aEEG is mainly used to study brain damage caused by neonatal asphyxia. However, there is no clinical basis for monitoring brain function and neurodevelopmental evaluation in children with ectopic growth retardation [3].

Various high-risk factors in preterm infants can increase the occurrence of asphyxia and increase the probability of brain damage and developmental abnormalities in preterm infants. Therefore, early detection of brain damage in preterm infants with asphyxia, accurate assessment of the degree of brain damage, reasonable assessment of the prognosis, guidance, and management of preterm infants will help them to pass the critical period of brain development smoothly and will greatly help reduce the disability caused by brain injury in preterm infants with asphyxia. Therefore, early detection and evaluation of brain damage in preterm infants with asphyxia has become the focus of attention. However, the current clinical diagnosis and evaluation of hypoxic-ischemic encephalopathy are mainly focused on full-term newborns. There is still no unified opinion on the diagnosis and treatment of brain damage in preterm infants caused by asphyxia. In particular, the lack of objective evaluation indicators has led to difficulties in early diagnosis and treatment, and the early neurodevelopment of preterm infants cannot be intervened and treated on time [4]. Furthermore, preterm infants themselves have a high risk of abnormal brain development. Brain development is in rapid growth, so it is particularly difficult to clinically seek objective evaluation indexes for preterm infants' brain function dynamic development. At present, the objective diagnosis and evaluation methods of brain injury and brain development mainly rely on imaging methods such as craniocerebral ultrasound and MRI, which are difficult to early dynamic monitoring due to technical limitations. In recent years, more and more studies have found that although EEG lacks specificity in diagnosing brain injury, it is one of the sensitive indicators for judging the state of brain function. Brain function damage usually precedes the damage of brain structure, so EEG can be used as an objective evaluation index of early brain damage and prognosis. However, due to electroencephalography and analysis technology problems, the clinical practice has not been widely developed. Therefore, seeking a simple and objective treatment for EEG dynamic monitoring is one of the current research focuses [5].

Due to the slow speed of paper feeding, adjacent waveforms are superimposed and integrated, which manifests as wide and narrow bands. The semilogarithmic coordinate means that the amplitude axis is expressed in a logarithmic coordinate. The primary purpose is to enable very low amplitude (<5 pv) background activities to be enhanced when displayed. Through the above process, the result obtained is no longer a conventional EEG signal but a spectral band signal representing the overall activity of the EEG background. Clinically, it is possible to classify EEG background waveforms through intuitive analysis of aEEG signals. The obtained background waveform types are indicators for the diagnosis and prognosis of encephalopathy [6], which directly reflect the brain function during the monitoring period. Compared with conventional EEG, on the one hand, due to the small number of aEEG electrodes, it is convenient for long-term recording. Therefore, it is especially suitable for bedside brain function monitoring of high-risk newborns in neonatal intensive care units (NICUs). On the other hand, aEEG is easy to operate, intuitive, and easy to analyze. At present, many studies have shown that there is good consistency between aEEG and conventional EEG.

## 2. Related Work

For nearly 20 years, aEEG has been utilized to monitor newborn brain activity, primarily for the auxiliary diagnosis of other encephalopathies in term neonates and assessing neurodevelopmental prognosis. It has excellent specificity and sensitivity, according to many investigations. First, AEEG was utilized to capture. It was found that aEEG can predict abnormal neurodevelopmental results with a specificity of 82%, a positive predictive value of 85%, and a negative predictive value of 100%. Second, the study pointed out that aEEG can diagnose encephalopathy within 6 hours after birth in neonates with perinatal asphyxia. Their positive predictive values are 86% and 84%, and they are 96% and 91%, respectively. Early research has shown that an EEG may aid in diagnosing encephalopathy and the prognosis of neurodevelopment in a short amount of time following birth. Literature [7] compared the characteristics of the early neurological examination and single-channel aEEG in diagnosing encephalopathy in 50 severe term neonates. The results show that abnormal aEEG has advantages over early abnormal neurological examinations in terms of specificity (89% vs. 78%) and positive predictive value (73% vs. 58%). When the two are combined, the highest specificity (94%) and positive predictive value (85%) can be achieved. The value of aEEG in the early diagnosis and prognosis of HIE has been confirmed by many studies. The aEEG and other reperfusion and reoxygenation parameters were investigated during newborn perinatal HIE and 2 hours later in literature [8]. The findings were compared to the relevant pathophysiological reactions in people.

It was found that the type of aEEG had the best correlation with the severity of neonatal HIE. This conclusion suggests that aEEG is a very sensitive indicator of HIE, which is very helpful for diagnosing HIE. Literature [9] shows that the background type of aEEG in the short term after birth asphyxia is highly correlated with the overall glucose metabolism of the brain. In addition, some studies have found that aEEG is another discriminant index for screening treatment subjects. Hypothermia is a commonly used treatment method for neonatal encephalopathy. Still, because treatment measures can produce more severe side effects, patients need to be strictly screened before treatment to determine that the benefits they can get from the treatment outweigh the harm. Literature [10] shows that a high negative predictive value (84%) of aEEG can avoid unnecessary harm to newborns during treatment. Literature [11] proved that neonates with asphyxia can use aEEG to screen whether they need neurological hypothermia therapy after birth, so that hypothermia therapy for children with encephalopathy may be performed within 6 hours after birth. These studies have shown that using aEEG monitoring for children with encephalopathy shortly after their birth can help screen children who are suitable for neurological treatment for timely treatment.

Previous aEEG studies have found that the background activities of deficient birth weight infants are mainly discontinuous and gradually become continuous with the increase of GA. In recent years, most studies on the use of aEEG to assess brain function in preterm infants have shown that the maturity of aEEG in preterm infants is related to GA. Literature [12] believed that the continuous increase of EEG background activity is related to the cortical folding process. Other researchers also believe that this continuous increase in brain electrical activity may be related to the development and maturation of excitatory synapses in the brain. Literature [13] used different definition standards to study preterm infants. The results show that GA 24-25 weeks of very low weight preterm infants mostly shows discontinuous low voltage mode (<3 uV), and 26-27 weeks of preterm infants shows discontinuous high voltage mode (3–51 aV). As the GA increases, the voltage gradually increases, and it changes to a continuous background mode. Literature [14] found that the aEEG abnormal detection rate changed rapidly within 2 weeks of PA for normal preterm infants in different GA groups, and the background continuity pattern of aEEG was significantly improved. The smaller the GA at birth is, the more it shows the “catch-up phenomenon” after birth. This phenomenon of continuous maturation of aEEG, which is significantly related to PA, speculates that extrauterine factors may promote the adaptive maturation of the brain of preterm infants. Preterm infants with lower GA may have accelerated brain maturation within 2 weeks after birth, suggesting that preterm infants are prone to brain development abnormalities and brain damage during this period. The results of a one-week aEEG monitoring experiment for deficient birth weight infants starting 12–48 hours after birth confirmed [15] that early aEEG examination within 1 week after birth can predict the poor prognosis of preterm infants. If it is combined with cranial ultrasonography, it can improve the sensitivity to the poor prognosis of preterm infants. The recent aEEGxg study showed that the appearance and stable presence of SWC in preterm infants is significantly related to the long-term average prognosis [16], and immature SWC can be identified in the background of healthy infants at about 26-27 weeks of pregnancy. GA develops into a mature SWC at 31-32 weeks, and SWC is easily recognized clearly due to the significant increase in bandwidth during the quiet sleep period. The evolution of SWC is one of the essential electrophysiological manifestations of brain maturation in preterm infants.

## 3. Materials and Methods

The study included 140 preterm infants who were hospitalized in the NICU of a hospital from January 2019 to December 2020 with a gestational age (GA) of less than 37 weeks who met the enrollment criteria and survived and followed up to the adjusted age of 12 months. All preterm infants were admitted to NICU within 1 hour after birth and received corresponding treatment in accordance with the “Guidelines for the Management of Preterm infants” compiled by the Chinese Medical Association. All preterm infants must meet the basic inclusion criteria and basic exclusion criteria. Basic inclusion criteria: preterm babies with birth weights appropriate for gestational age, and preterm infants who have not used sedatives or neuroactive medications for at least 48 hours prior to the study. The asphyxia and normal groups must still satisfy their respective entrance and exclusion criteria. Basic exclusion criteria are as follows: chromosomal diseases or congenital developmental abnormalities; family genetic disease history; intrauterine infection; intracranial hemorrhage caused by head trauma; a body temperature of less than 34 degree Celsius; preterm babies whose legal guardian refuses to participate in the study and follow-up; and preterm babies who did not complete continuous aEEG monitoring, imaging examination, or postnatal follow-up. Normal group exclusion criteria: any of the following abnormalities found in clinical or aEEG monitoring, analysis, and head imaging examinations: convulsions or seizures (based on clinical convulsions and/or a complete 8-lead aEEG diagnosis made by a professional pediatric neurologist), grade III-IV intraventricular hemorrhage (IVH) (Papile classification), cystic periventricular leukomalacia, congenital diseases, and preterm infants with local areas that are not suitable for electrode placement (such as cannon skin lesions or intracranial hydrops that drainage).All children completed head ultrasound examination within the first week after birth and were reviewed weekly. If intracranial hemorrhage is confirmed, at least one head CT or MRI examination should be completed within 3 weeks of PNA to exclude periventricular white matter softening, or imaging examination should be selected according to the clinical symptoms [17].

This paper analyzed the diagnosis and prediction effect of amplitude eukaryotic EEG by setting the control and test groups. Among them, the control and experimental groups are 70 people, and the two groups of newborns have no statistical significance in all aspects of the parameters, so that the experimental study can be carried out.

The experiment uses Nicoletone EEG (which contains conventional EEG recordings, convertible amplitude integration EEG, frequency band energy map, and envelope map mode) from Nicolet Company in the United States. In the experiment, the 12-lead scalp electrodes (F3, F4, T3, T4, T5, T6, C3, C4, P3, P4, O1, and O2) are placed according to the 12.5–25 system recommended by the American Neurophysiological Association. The reference electrode is pasted between FZ and CZ, and the silver electrode on the plate is fixed on the corresponding scalp with conductive paste, and the surgical mesh cap is used to strengthen the fixation. At the same time, the experiment added 3 pairs of physiological parameter records, including ECG leads (applied to the chest of the child), mandibular muscle electrical leads (applied to the child's mandible or masseter muscle), left and right eye movement leads (attached to the left and right eyes diagonally above, diagonally above the right side, or diagonally below the left side, and diagonally above the right side). In the experiment, the children are selected to be born 3–7 days, the average initial monitoring time is 4.72 ± 1.55 days, and continuous bedside EEG monitoring is performed. One monitoring time is 12–20 hours, and the average monitoring time is 15 ± 2 hours. Thus, the CEEG record contains at least one complete sleep cycle. The monitoring of CEEG is carried out at nighttime when there is less medical operation and interference.

The baby is placed in an incubator. After feeding, the premature baby is placed in a quiet environment and connected to aEEG electrodes. aEEG is a simplified single-channel EEG monitoring, and the electrodeposition is equivalent to P3 and P4 of the 10/20 international electrode placement method. The reference electrode is located on the frontal midline, 25 mm forward from the center of the head. The EEG signal in the semilogarithmic form is traced, and the waveband pattern is traced in the form of amplitude at the same time. The monitoring time lasts for 6 hours, and the nursing operation and feeding time are concentrated in a short period of time.

Preterm infants in each group are monitored by bedside craniocerebral ultrasound every week after birth. The experimental counts of each child's gestational age, birth weight, hospitalization time, and weight began to decline at the age and fell to the lowest age. Moreover, the experiment measures the percentage of birth weight when the body weight drops to the lowest, the milking time, and the age when the milk is needed for growth. In addition, the experiment recorded the number of anemia and infections in each group of infants during their hospitalization, and the number of preterm infants who needed blood transfusions [18].

When the gestational age of the premature baby is 40 weeks or the premature baby is discharged from the hospital for 1 month, the Philips InteraAchieva 3.0 superconducting MR instrument is used for craniocerebral nuclear magnetic examination. At the time of discharge in 6 months, the pediatric care department is followed up to observe feeding, weight gain, etc. and is evaluated by GESELL. Normal children are ≥85 points, boundary children are 75∼85 points, <75 points are abnormal children, suggesting that motor development is lagging, and brain injury is considered.

All newborn BAEP examinations are performed within 24 hours after blood draw. The experiment is carried out with the Nihon Kokoh 9204k EMG instrument. During the examination, the surrounding environment should be kept quiet, and appropriate light, temperature, and humidity should be provided to ensure that all newborns are calm. Those who are not cooperating, such as crying and restlessness, etc., should be given 10% chloral hydrate (50 mg/kg) retention enema to calm down and fall asleep. Before the inspection, the external ear canal is cleansed, and the sebum on the skin where the electrode is put is removed using a wipe gel. The ground electrode is positioned between the forehead and the brows, the recording electrode is placed on both sides of the mastoid, the reference electrode is placed on the head, the electrode impedance cannot exceed 5kO, and the bandpass filter is between 100 and 3000 Hz. Earmuffs are used to provide polar wave-shrinking stimulation to both ears at an intensity of 80 dB, a frequency of 10 Hz, a superimposition rate of 2000 times per minute, and duration of 10 ms. Before the test, the researchers used BAEP to determine the hearing threshold and gradually raised the stimulus intensity low to high. The hearing threshold is the lowest intensity that caused the *v* wave to emerge.

Those with average auditory response threshold continue to complete various BAEP examinations. Each ear is tested for two rounds for better repeatability. For nonresponders, the stimulation intensity can be increased up to 100 dB to record the best BAEP waveform. Experienced full-time competent technicians carry out all operations and results of analysis.

The experiment uses SPSS 16.O software for statistical analysis, and the measurement data is expressed as mean ± standard deviation ± *s*.The comparison of the means of two independent samples accords with the data of normal distribution and homogeneity of variance, and the *t*-test is used. For those with nonnormal distribution and uneven variance, the nonparametric rank-sum test is used. The chi-square test is used to compare the count data between groups. *P* < 0.05 indicates that the difference is statistically significant [19].

## 4. Results

This article mainly studies the prediction effect of amplitude-integrated EEG on the brain damage and long-term nervous system development of late preterm infants. The effect is verified by designing controlled experiments and statistical methods. Moreover, this paper evaluates the real-time monitoring effect and short-term prediction effect of amplitude-integrated EEG on brain damage of preterm infants and the prediction effect of long-term nervous system development and counts evaluation results.

This article counts the monitoring effect of amplitude-integrated EEG on the brain damage of late preterm infants and compares it with the traditional monitoring effect of brain damage of late preterm infants. The results are shown in Table 1 and Figure 1.

From the above comparison, amplitude-integrated EEG monitoring effect on brain injury of late preterm infants is significantly better than traditional monitoring methods. After that, this paper evaluates the effects of long-term nervous system development of late preterm infants. The results are shown in Table 2 and Figure 2.

From the above comparison, the effect of amplitude-integrated EEG on the evaluation of the recent nervous system development of late preterm infants is significantly better than that of traditional monitoring methods. After that, this paper detected the effect of amplitude-integrated EEG on late preterm infants' long-term nervous system development. The results are shown in Table 3 and Figure 3.

Through experimental analysis, it can be seen that the amplitude-integrated EEG is very effective in predicting the long-term nervous system development of late preterm infants.

## 5. Conclusion

The incidence of preterm infants continues to rise, and the survival rate of preterm infants is getting higher and higher. What follows is that the problem of brain damage in preterm infants is getting more and more attention. Almost 25% of young preterm infants have potential neurodevelopmental problems, while full-term infants account for only 4%. Among surviving small preterm infants, the incidence of cerebral palsy increased significantly with the decrease of gestational age at birth. The results of this study are also consistent with this. Asphyxia is the main cause of perinatal death and poor neurological prognosis. Due to the possible pathological conditions of the pregnant mother and this kind of premature infant, various perinatal abnormalities are prone to occur, of which perinatal asphyxia is one of the most common diseases. The incidence of hypoxic-ischemic encephalopathy (HIE) caused by asphyxia has continued to rise in the past 40 years. Various high-risk factors in preterm infants can increase the incidence of asphyxia and increase the probability of brain damage and developmental abnormalities. Early detection of brain damage in premature infants with asphyxia and accurate assessment of the degree of brain damage are important. The management of preterm infants can help them smoothly past the critical period of brain development, which will significantly help reduce the disability caused by brain injury in premature infants with asphyxia. In the past few decades, due to the development of brain protection therapy for asphyxia after birth, it has become possible to reduce delayed neuronal death and programmed cell death. However, the precise time window of brain protection therapy is still unclear. Because this treatment may have serious side effects, clinicians need to strictly evaluate and select newborns who have benefited from the treatment before it can be recommended. Therefore, it has important clinical significance to explore the early accurate auxiliary diagnostic indicators. Some previous studies have found that some early neonatal monitoring parameters such as fetal heart monitoring, umbilical artery blood PH value, and Apgar score, whether alone or in combination, have minimal clinical guidance value. However, conventional EEG is the gold standard for electrophysiological evaluation of brain function. The 8-lead EEG placed according to the international 10–20 system is a sensitive method for diagnosing neonatal convulsions and evaluating the background characteristics of neonatal EEG.

Studies have found that neonatal EEG patterns, such as continuity, particular EEG waveforms, and SWC, change with different GAs. For the research of neonatal EEG physiological maturity, current scholars mostly use multilead EEG recording. Studies have confirmed that the use of CEEG for neuroelectrophysiological monitoring may be a very clinically valuable means of evaluating brain function within 24 hours after birth. aEEG is a clinical EEG monitoring technology for neonates developed in recent years. It is a simplified, single-lead EEG physiological monitoring that can reflect changes in background activities and epileptiform activities. Moreover, it has the characteristics of simple operation, less environmental interference, straightforward interpretation, long-term continuous bedside monitoring, and can be used for brain function monitoring of various high-risk newborns. Therefore, applying aEEG for continuous brain function monitoring has become a part of daily monitoring in neonatal intensive care units abroad. As the use of aEEG in the NICU becomes more and more common, the results of several studies on asphyxiated term neonates show that aEEG is a valuable technical means for early assessment of long-term prognosis within 6 hours after birth.

In this paper, experimental studies have proved the prediction effect of amplitude-integrated EEG on brain damage and long-term nervous system development in late preterm infants, which provides a good foundation for subsequent clinical diagnosis and treatment strategies.

## Figures and Tables

**Figure 1:** Statistical diagram of the effects of real-time monitoring of brain damage in late preterm infants.

**Figure 2:** Statistical diagram of the evaluation effect of amplitude-integrated EEG on the recent nervous system development of late preterm infants.

**Figure 3:** Statistical diagram of the evaluation effect of amplitude-integrated EEG on the long-term nervous system development of late preterm infants.

**Table 1:** Statistical table of the effects of real-time monitoring of brain damage of late preterm infants.

Num	Control group	Test group	Num	Control group	Test group	Num	Control group	Test group
1	90.4	98.9	25	91.7	94.7	48	89.3	94.1
2	88.7	98.1	26	89.4	97.8	49	92.3	97.2
3	89.0	94.2	27	88.6	96.1	50	93.8	95.6
4	93.8	98.6	28	88.2	95.9	51	90.3	97.6
5	88.5	98.6	29	92.7	98.7	52	91.9	94.9
6	88.6	97.7	30	91.8	98.5	53	93.6	96.7
7	91.2	95.5	31	91.2	98.5	54	92.5	95.2
8	93.0	95.6	32	90.3	96.0	55	88.2	94.2
9	90.7	98.9	33	88.9	95.0	56	88.4	94.0
10	89.7	97.0	34	89.8	98.8	57	93.0	95.7
11	91.9	98.5	35	91.8	96.1	58	93.7	94.2
12	88.7	97.9	36	88.5	95.7	59	91.1	94.7
13	89.3	98.9	37	90.5	97.7	60	93.0	96.4
14	90.7	95.4	38	89.1	98.7	61	91.0	97.6
15	92.8	95.7	39	91.1	95.9	62	92.9	96.1
16	93.8	95.2	40	89.1	97.1	63	89.1	97.9
17	91.6	95.1	41	92.9	96.6	64	92.0	95.5
18	93.8	94.9	42	90.6	95.6	65	90.7	94.4
19	90.3	98.7	43	90.7	98.2	66	92.4	94.5
20	93.9	97.3	44	93.1	95.1	67	93.6	95.0
21	90.7	97.7	45	91.7	94.5	68	90.2	97.6
22	90.4	97.3	46	91.2	95.1	69	92.0	99.0
23	92.6	95.1	47	91.9	96.4	70	92.5	94.0
24	89.0	96.9						

**Table 2:** Statistical table of the evaluation effect of amplitude-integrated EEG on the recent nervous system development of late preterm infants.

Num	Control group	Test group	Num	Control group	Test group	Num	Control group	Test group
1	86.2	88.5	25	78.4	91.3	48	80.4	91.5
2	78.5	91.0	26	78.6	89.0	49	88.2	88.6
3	78.9	90.3	27	82.4	84.3	50	85.0	89.1
4	88.0	88.1	28	84.8	87.5	51	84.2	84.9
5	79.7	85.5	29	88.9	91.6	52	82.3	88.4
6	84.4	83.8	30	84.3	84.0	53	85.1	88.5
7	80.0	88.1	31	85.5	83.4	54	79.5	87.4
8	86.1	85.1	32	85.7	86.9	55	86.8	90.1
9	85.3	90.3	33	87.8	85.0	56	81.6	88.2
10	88.8	89.4	34	86.3	91.8	57	83.6	90.1
11	79.3	84.3	35	82.8	89.8	58	85.6	88.1
12	87.0	85.9	36	80.2	85.1	59	84.2	83.9
13	88.4	88.7	37	81.5	85.1	60	78.4	86.2
14	83.3	90.0	38	82.0	86.5	61	86.4	84.6
15	85.4	87.9	39	87.3	91.0	62	79.8	87.0
16	82.8	90.9	40	88.6	90.0	63	85.1	85.1
17	83.9	83.6	41	84.3	89.3	64	86.4	87.6
18	78.5	88.9	42	81.8	83.1	65	84.8	86.5
19	88.8	91.0	43	80.2	90.0	66	82.7	85.4
20	88.3	89.1	44	84.4	87.0	67	85.0	84.7
21	79.4	84.9	45	84.5	90.1	68	83.2	90.9
22	87.3	89.1	46	85.1	86.6	69	87.9	87.6
23	87.0	85.5	47	83.7	83.6	70	78.9	88.2
24	88.4	91.8						

**Table 3:** Statistical table of the evaluation effect of amplitude-integrated EEG on the long-term nervous system development of late preterm infants.

Num	Control group	Test group	Num	Control group	Test group	Num	Control group	Test group
1	76.3	81.8	25	81.1	83.2	48	80.0	82.4
2	83.4	86.1	26	76.3	86.7	49	80.1	90.6
3	84.9	87.0	27	80.5	83.0	50	83.0	87.2
4	76.1	83.7	28	76.3	83.0	51	76.9	86.3
5	76.5	88.4	29	80.8	83.1	52	77.1	88.9
6	78.9	84.9	30	83.7	87.0	53	83.6	84.4
7	84.2	82.7	31	82.9	82.6	54	82.6	86.6
8	76.2	86.6	32	77.9	85.9	55	81.6	86.0
9	81.0	86.7	33	80.1	82.1	56	78.6	86.7
10	76.4	81.1	34	77.8	83.9	57	77.0	84.6
11	84.1	87.6	35	84.3	86.3	58	82.2	87.5
12	79.7	85.9	36	76.8	88.9	59	80.0	86.6
13	82.7	86.9	37	80.6	82.9	60	79.5	88.9
14	76.1	85.7	38	79.7	87.8	61	84.0	87.1
15	81.7	83.8	39	80.4	83.8	62	78.8	86.7
16	83.2	89.0	40	84.9	87.9	63	83.1	83.4
17	76.9	86.9	41	81.3	85.3	64	79.9	81.5
18	76.0	85.6	42	84.8	87.2	65	78.2	85.5
19	80.0	87.8	43	80.0	85.1	66	83.6	84.2
20	76.6	87.9	44	76.4	85.5	67	80.6	89.0
21	79.8	85.2	45	81.8	81.5	68	80.7	87.3
22	80.4	86.3	46	82.4	82.3	69	84.1	86.8
23	84.5	88.7	47	80.1	85.5	70	83.2	84.9
24	85.0	85.2						

## Data Availability

The data used to support the findings of this study are included within the article.
